# CT Imaging Characteristics and Influence Factors of Renal Dialysis-Associated Peritoneal Injury

This article has been retracted.

**DOI:** 10.1155/2021/5591124

**Published:** 2021-04-20

**Authors:** Jin Tong, Wangda Xu

**Affiliations:** ^1^Department of Nephrology, Zhuji People's Hospital, Zhuji, Zhejiang 311800, China; ^2^Zhejiang Chinese Medical University, Hangzhou, Zhejiang 310053, China

## Abstract

Peritoneal dialysis (PD), as one of the main renal replacement modalities for end-stage renal disease, gets the advantages of better protection of residual renal function and better quality of survival. However, ultrafiltration failure after peritoneal injury is an important reason for patients to withdraw from PD treatment. Peritonitis is a major complication of peritoneal dialysis, which results in an accelerated process of peritoneal injury due to direct damage from acute inflammation and local release of cytokine TGF-*β*. In this paper, the application of ultrasound to examine the peritoneum revealed a positive correlation between peritoneal thickness and the development of peritonitis. The results of this study also further confirmed the effect of peritonitis on peritoneal thickening. A multifactorial regression analysis also revealed that peritonitis and its severity were independent risk factors for peritoneal thickening and omental structural abnormalities. This paper reported a correlation between mural peritoneal thickness and peritoneal transit function. In this study, patients with high peritoneal transit and high mean transit were found to be more prone to omental structural abnormalities than patients with low mean and low transit and a higher proportion of patients with mural peritoneal thickening, but this did not reach statistical significance, which may be related to the still small number of cases.

## 1. Introduction

End-stage renal disease (ESRD) is the end-stage of chronic kidney disease (CKD), characterized by high incidence, critical illness, high medical costs, poor prognosis, and high socioeconomic burden [1–5], and has become an important public health problem worldwide. The prevalence of CKD is 14.8% in the United States and 10.8% in China [6]. Between 1990 and 2013, global life expectancy increased by approximately 5.8 years, while CKD significantly reduced life expectancy by 0.1 years [7]. By 2040, CKD will be ranked 5^th^ in terms of reduction in life expectancy, up from 16^th^ in 2016, which shows its harmful effects. Between 1990 and 2016, the global risk of CKD increased significantly, with an 89% increase in morbidity, a 98% increase in mortality, and a 63% increase in disability-adjusted life years (all healthy life years lost to premature death and disability from all diseases) [8], with $114 billion spent annually on CKD in the United States [9].

As a result, ESRD will create a serious socioeconomic burden worldwide. Alarmingly, even with regular nephrology follow-up of these ESRD patients, more than 60% of newly diagnosed ESRD patients are unplanned when starting renal replacement therapy [10] and often require emergency initiation of dialysis [11], although emergency initiation of dialysis is the preferred mode of initiation, it is still a common problem worldwide. Although it is the preferred mode of initiation, urgent initiation of dialysis is still a common problem worldwide, accounting for 30–50% of patients starting dialysis [12]. Ultrasound is a noninvasive imaging method, but because it has mostly similar echoes in the differential diagnosis of benign and malignant renal tumors and the differential diagnosis is highly correlated with the physician's subjective diagnosis [13]. The use of ultrasound contrast peak time, intensity, and mode of enhancement to identify benign and malignant renal tumors and RAMLwvf with cc RCC has also been studied quite a bit, and the previous authors used the mode of enhancement of contrast agent within the mass to identify benign and malignant renal tumors, although its sensitivity and specificity were above 0.9 and found that small-sized benign renal tumors mostly showed homogeneous enhancement and homogeneous fading, but although its sensitivity and specificity were above 0.9 and it was found that benign renal tumors of small size mostly showed homogeneous enhancement and homogeneous fading, its diagnostic features in larger benign renal masses were not obvious and insufficient to differentially diagnose benign and malignant renal tumors; Alkatout used contrast-enhanced ultrasound to identify the relative peak time and relative mean transit time of contrast agent in RAMLwvf and cc RCC, and the difference between their values was not very obvious [14] and could not be promoted in clinical application; some people used ultrasound imaging contrast to diagnose benign and malignant renal tumors. CT is the initial method used to identify benign and malignant renal tumors, and CT perfusion scan is a noninvasive method to predict the blood supply to the tumor, which is more reliable in identifying benign and malignant renal tumors. Although it can better reflect renal hemodynamic changes, as shown in Figure 1, CT perfusion postprocessing is cumbersome, and the difference between its values is not obvious, in addition, the concentration of contrast agent varies greatly depending on the operator, which largely limits its clinical application [15]. Energy-spectrum CT with iodine as the base material has a prominent and magnifying effect on the display of masses with a rich blood supply of lesions using energy-spectrum parameters of different renal benign and malignant tumors, such as iodine (water) base map and iodine (water) scatter map to analyze the differences [16]. In the solid part of different lesions, there are also studies using energy spectrum CT to analyze the iodine concentration of the mass and the standardized iodine concentration, etc., and good diagnostic results have been achieved [17–19].

In this paper, we investigated that iodine basal value is a quantitative parameter with high accuracy and can directly reflect iodine uptake in organs and tissues, which provide effective support for its application to benign and malignant renal tumors. The IC and NIC of enhanced cortical and medullary stage cc RCC are higher than RAMLwvf, and the difference is statistically significant, suggesting that iodine content is related to the biological characteristics and pathological structure of renal tumors. This is related to the fact that malignant renal tumors have more neovascularization than benign tumors, and most of them are not mature vessels with large endothelial gaps, so cc RCC has high vascular permeability and rapid contrast extravasation. Therefore, the iodine content is high, while RAMLwvf has slow growth, with relatively few neovascularization and relatively mature vessels, and low vascular permeability, so the iodine content of the lesion is lower. Although its sensitivity and specificity are high, the differences between the iodine base values are not obvious and there are many overlaps, so its application in clinical practice continues to be questionable. Normal peritoneum is invisible or faintly visible on computed tomography (CT) scans of the abdomen, but with the prolongation of dialysis age and the effect of peritonitis, peritoneal imaging changes can be seen on CT of the abdomen in some patients, but the pattern of changes is still unclear. The purpose of this paper is tantamount to analyze the changing pattern of imaging features of peritoneal injury and its influencing factors.

## 2. Related Work

MR imaging performance and DWI differentiation MRI is useful for diagnosing cc RCC and RAMLwvf, and chemical shift imaging sequences can evaluate the fat content in voxels. cc RCC and RAMLwvf with poor differential diagnostic accuracy; researchers explored the chemical shift signal intensity index (CS-SII) in discriminating cc RCC from RAMLwvf, but its difference between the two was not statistically significant [20]. In addition to conventional MRI sequences, several functional MRI imaging examinations have been performed: contrast-enhanced MRI scanning techniques, arterial spin labeled perfusion imaging (ASLPI), magnetic resonance contrast-enhanced MRI scans using GD-DTPA, and a contrast agent metabolized by the kidneys can cause some damage to the kidneys and limit their use in renal cancer patients with renal insufficiency. The study of MRS and blood oxygen level-dependent MR imaging for kidney cancer has many technical limitations, and its imaging is affected by age and kidney function level, and the study of this aspect is still immature.

ASLPI was first used as a measure of blood perfusion in brain tissue and is being explored in normal kidney and renal tumors [21]. A comparative study using the latest IVIM sequence of magnetic resonance diffusion-weighted imaging and the differential diagnosis of benign and malignant renal tumors has enabled the diagnosis of magnetic resonance to be elevated to the histological level, and the lesions can be studied quantitatively, not only to derive the corresponding parameter ranges of normal renal parenchyma and benign and malignant renal tumors but also to identify benign and malignant renal tumors using the IVIM sequence with AUC values, sensitivity, and specificity of 0.7. The sensitivity and specificity were about 0.7, and the values were low. Histopathological confirmation of renal cell carcinoma has been performed by heterogeneity analysis (mean, standard deviation, skewness, and kurtosis) of intravoxel incoherent motion imaging (IVIM) parameters (perfusion fraction (fp), tissue diffusion coefficient (Dt), and pseudodiffusion coefficient (Dp)) in 44 patients who underwent preoperative DWI MRI. However, due to the low spatial resolution of IVIM images, the normal renal cortex and tumor borders cannot be clearly identified, which makes the measurement work very difficult and there are some errors in the measurement results. DWI is a magnetic resonance functional imaging technique based on the diffusion motion of water molecules in the living body, and with the application of MRI ultrafast imaging sequences, especially planar echo imaging sequences, DWI has been gradually applied to abdominal imaging diagnosis. The kidney is located in the retroperitoneal space and is relatively unaffected by respiratory motion, and the same satisfactory image quality can be obtained with free breathing as with breath-holding [22–24]. DWI signal intensity mainly reflects the tissue structure, nucleoplasmic ratio, distribution of water molecules inside and outside the cells, cell density, and so forth. A large number of studies have shown that ADC values are higher in benign tumors than in malignant ones, cystic tumors than in solid tumors, and necrotic areas than in nonnecrotic areas. A number of studies have shown that ADC values are valuable in the differential diagnosis of benign and malignant tumors in the kidney, and differentiating benign tumors from malignant tumors may reduce inappropriate nephrectomies. False ADC (Dp), true ADC (Dt), and perfusion fraction (fp) were calculated from diffusion-weighted images using mono- and biexponential models. ADC values for RAMLwvf were significantly lower than those for cc RCC, and the biexponential diffusion decay model ADC was able to reflect diffusion more accurately than the monoexponential diffusion decay model.

Unlike traditional empirical routine analysis based on visual recognition, “imaging histology” refers to the high-throughput extraction of quantitative features from a large number of images, which enables the conversion of images to large amounts of data and the construction of histological labels to comprehensively characterize the subtleties of lesions and thus assist in clinical decision-making. These quantitative features are obtained from individual imaging data such as US, CT, MR, and PET-CT through a large number of algorithms, which can reflect the physiological heterogeneity of the mass in the region of interest, thus revealing a series of information that cannot be detected by the naked eye related to pathological type, molecular typing, treatment response and prognosis.

## 3. Enhanced CT for Kidney Injury Detection

### 3.1. Imaging Histological Features

Image histology features are classified as follows: shape features, first-order histogram features, second-order histogram features, or texture features; the basic principle is to select different statistics to extract statistical features of the original image or parameter map. The statistical parameters of the statistical method are divided into first-order, second-order, and higher order. The first-order statistics describe the features related to the intensity distribution of voxels within the ROI, and the method is based on the grayscale histogram, and the features include the mean, median, minimum, maximum skewness, and kurtosis; the second-order statistics describe the features of the intensity level of the spatial distribution of voxels and apply the spatial grayscale dependence method or covariance matrix, by calculating the correlation between one pixel and another pixel in the image at a certain distance and direction and depicting the image in the direction of spatial grayscale. It is a synthesis of visual perceptual image features and reflects the local texture characteristics. The second-order parameters include the grayscale cooccurrence matrix and grayscale level length matrix. The higher order is the application of adjacent pixel gray level difference matrix, which reflects the intraregional intensity variation or the distribution of homogeneous regions. The use of imaging histology is expected to be a precise diagnosis method for cancer diseases, which is of great value for the selection of clinical surgical modalities and prognosis. In today's world of precision therapy, the accuracy of this prediction system for individualized prediction is limited and can be derived from the following equation:

(1) $$\begin{array}{c} g_{i}=|{\text{User}}_{i}:k_{1},k_{2},\ldots k_{i}\rangle . \end{array}$$

Therefore, there is a clinical need for more accurate predictive models to achieve precise and individualized assessment. Imaging histology has made great progress in improving techniques for prognostic assessment of tumors and selection of cancer treatments. Textural characteristics of 87 metastases before and after two cycles of tyrosine kinase inhibitor treatment were analyzed by the following equations, which revealed a 3%–45% reduction in entropy and 5%–21% improvement in consistency parameters of metastases after two cycles of TKI treatment, using COX regression analysis to assess textural characteristics, and response evaluation criteria for solid tumors:

(2) $$\begin{array}{c} g_{i}=\left\{{\text{guest}}_{i},\ldots ,{\text{guest}}_{q}\right\},\\ g\text{set}=\left({\text{CTvalue}}_{1},\ldots ,{\text{CTvalue}}_{i}\right). \end{array}$$

While there was no statistical difference in texture characteristics between the groups with and without regional lymph node metastasis, it was concluded that texture analysis could be an effective diagnostic method to predict the site of cc RCC metastasis. The above equations confirm the value of imaging histology in prognosis prediction, efficacy evaluation, and long-term monitoring of kidney cancer, providing an efficient and feasible way to achieve precision medicine.

There are likewise many studies on the differential diagnosis of renal tumors in imaging histology. The aforementioned authors retrospectively analyzed 460 cases of cc RCC imaging data and found that the histological model established by them is a reliable predictor in identifying both high- and low-grade cc RCC. It has obvious advantages over biopsy, which not only reduces the pain caused by biopsy but also improves work efficiency, reduces the financial burden on patients, and provides a healthier and safer way to review the patient's condition in the future. In comparing three time-phase CT images with conventional CT analysis (border, cystic necrosis, and pseudo-envelope) by constructing a radiomics-based logistic classifier to identify cc RCC and RAMLwvf, it was found to have better diagnostic efficacy than conventional CT, with an AUC value of 0.95, which is higher than the results of this study. However, its small number of screened cases is also one of the reasons for its better results. In a multi-institutional dataset, using conventional MR imaging, deep learning can noninvasively identify benign renal tumors and renal cancer with accuracy, sensitivity, and specificity comparable to expert and radiomics, with an accuracy smaller than the present study. Some have used the value of MRI texture parameters in the differential diagnosis and histological grading of cc RCC versus non-cc RCC with AUC values greater than 0.8, in addition to progress in predicting lymph node metastasis in other diseases, and histological features of biomarkers to predict survival.

### 3.2. Kidney Malignancy Damage Detection

Imaging genomics has also been studied in renal malignancies, where genes are determinants of tumorigenesis and understanding the microstructure of tumors can help in clinical tumor diagnosis, prognosis, and development of predictive biomarkers. Several recent studies have shown that, in cc RCC, in addition to inactivating mutations in VHL tumor suppressor genes, genes such as BAP1, PBRM1, SETD2, and KDM5C play a role in tumor development, for example, causing mutations in the ubiquitin-mediated protein hydrolysis pathway (UMPP) in cc RCC; recent sequencing studies of cc RCC sequencing studies have recently identified chromatin modification genes such as PBRM1, KDM6A/UTX, KDM5C/JARID1C, SETD2, MLL2, and BAP1 that are highly associated with inactivating point mutations in their progression and poor prognosis. Imaging genomics can be combined with artificial intelligence to extract tumor imaging features, at the same time, linking the genomic features to the potential mutation status of the tumor to achieve pretreatment prediction of tumor mutation status, while providing a therapeutic basis for clinically targeted drugs. Mutations in VHL were found to be associated with well-defined tumor borders, nodular tumor enhancement, and the presence of intratumor vasculature, while mutations in BAP1 and KDM5C were highly associated with infiltration of renal veins, with significant differences between solid cc RCC genotypes and cystic cc RCC genotypes and with no mutations in SETD2, KDM5C, and KDM5C in cc RCC genotypes. Mutations in SETD2, KDM5C, and BAP1 were absent in cc RCC genotypes, while mutations in VHL and PBRM1 were more common. Another study using imaging features correlated with mutational status (VHL, BAP1, PBRM1, SETD2, and MUC4) found that BAP1 mutations were associated with indistinct tumor borders and the presence of calcification, while MUC4 mutations were associated with an exophytic growth pattern of the tumor.

The study constructs an alternative imaging genomics-based model for the molecular detection of multiple gene expression in cc RCC (SOMA) by using CT imaging features, which uses microarray data and an image array of 28 features to evaluate each CT image with multiple regression for gene expression analysis, as shown in Figure 2. The predictive power of SOMA was then prospectively validated in an independent dataset, allowing for noninvasive independent prediction to assess patient survival and patient staging, and although current imaging genomics studies only correlate certain macroscopic image features with gene expression in RCC, this predicts that we can use artificial intelligence to extract high-throughput features on images and learn from the features. This will allow us to use imaging genomics features to predict the EGFR and Ki-67 expression levels and prognosis of low-grade gliomas, and to discover more features related to RCC gene expression, so that we can use images to predict the gene expression of RCC before surgery and implement individualized treatment for RCC patients to achieve the purpose of precision treatment.

## 4. Renal Dialysis and Injury Correlation

### 4.1. Emergency Initiation of Renal Dialysis (PD)

Urgent-start peritoneal dialysis (Urgent-start PD) is defined as ESRD patients requiring dialysis treatment within 14 days without permanent dialysis access, and peritoneal dialysis is used as the starting dialysis modality, as shown in Figure 3. The vast majority of ESRD patients referred late, who do not yet have dialysis access and require urgent initiation of dialysis, absolute contraindications, include the following: (1) chronic persistent or recurrent abdominal infections or extensive metastases from intra-abdominal tumors causing extensive peritoneal fibrosis and adhesions in the patient, reducing the dialysis area, affecting fluid flow in the peritoneal cavity, and causing diminished or lost peritoneal ultrafiltration function and reduced solute transport efficacy; (2) patients with severe skin disease, extensive abdominal wall infection, or extensive abdominal burns without a suitable site for PD catheter placement; (3) mechanical problems that are difficult to correct, such as surgically irreparable hernias, umbilical protrusions, and ventral fissures, which affect the effectiveness of peritoneal dialysis or increase the risk of infection; (4) severe peritoneal defects; and (5) patients with mental impairment and no suitable caregiver. Urgent-relative contraindications to start PD include the following: (1) serum potassium >6.5 mmol/L; (2) extremely elevated blood pressure; (3) severe volume overload with pulmonary edema; (4) uremic pericarditis or colitis; and (5) those with significant uremic symptoms.

Most studies have concluded that the incidence of bacteraemia is lower in patients with ESRD on emergency initiation of dialysis compared to HD and that long-term patient survival is not lower than that of patients on emergency initiation of HD. 123 patients on emergency initiation of dialysis were retrospectively studied, 66 in the PD group and 57 in the HD group, with a mean follow-up of 4.72 months. The results showed that the incidence of bacteraemia was significantly lower in the PD group than in the HD group, that patient survival was the same in the PD group compared with the HD group, and that emergency-start PD was not an independent risk factor for survival compared with emergency-start HD. A prospective study by Lobbedez et al. included 60 patients with emergency start dialysis, 26 in the Urgent-start HD group and 34 in the Urgent-start PD group, who started dialysis at an average of 4 days after placement in the Urgent-start PD group, with survival rates of 90% and 88% at 6 months and 1 year, respectively, and peritonitis-free survival at 6 months and 1 year. The 1-year survival rates for patients in the PD and HD groups were 78.9% and 82.9%, respectively, with no statistical difference.

### 4.2. Peritoneal Imaging Presentation

Abdominal CT scans revealed mural peritoneal thickening in 70 patients (64.22%), abnormal omental structure in 63 patients (57.80%), calcification of mural peritoneum and omentum in 4 patients (3.67%), abdominal compartment and encapsulated fluid in 11 patients (10.09%), and intestinal dilatation and obstruction in 24 patients (22.02%). Stratified by dialysis age, the proportion of wall peritoneal thickening and abnormal omental structure was significantly higher in patients with dialysis age >5 years than in patients with dialysis age <1 year (*χ*^2^ = 3.855, *P* = 0.050); stratified by the number of occurrences of peritonitis, the proportion of wall peritoneal thickening and abnormal omental structure was significantly higher in patients with more than 1 occurrence of peritonitis than in patients without peritonitis. In a stratified analysis based on total sugar intake, the proportion of patients with cumulative sugar intake >165 kg of abnormal omental structure was significantly higher than that of patients with cumulative sugar intake <60 kg (*χ*^2^ = 8.197, *P* = 0.004); in analysis by type of peritoneal transport, the proportion of omental structural abnormalities was significantly higher in patients with high peritoneal transport or high mean transport than in patients with low peritoneal transport or low mean transport (*P* < 0.05). Patients with low peritoneal transit or low mean transit (*P* < 0.05) are as detailed in Figure 4.

Logistic univariate regression analysis showed that the numbers of occurrences of peritonitis and cumulative peritonitis score were risk factors for peritoneal thickening. Age on dialysis, number of peritonitis episodes, cumulative peritonitis score, total sugar exposure, and high transit/high mean transit were risk factors for abnormal omental structure. Logistic multifactorial regression analysis showed that the numbers of peritonitis episodes and cumulative peritonitis score were independent risk factors for peritoneal thickening and abnormal omental structure; see Figure 5. The most important pathologic feature of peritoneal injury is the absence of an extensive mesothelial layer, with thickening of subcutaneous tissue and neovascularization. Peritoneal biopsy is a confirmatory method for the diagnosis of peritoneal injury, but it is an invasive procedure that is difficult to promote in the clinic and to observe dynamically. The sensitivity and specificity of biological markers related to peritoneal injury, such as transforming growth factor-*β* (TGF-*β*) and interleukin-6 (IL-6), are still uncertain and are still being explored. Therefore, early detection of peritoneal injury is still difficult, and there is a lack of specific indicators that can be observed dynamically.

## 5. Results and Discussion

Previous studies have analyzed the abdominal imaging features of patients with encapsulating peritoneal sclerosis by abdominal CT. There are no reports on the application of CT imaging to assess early peritoneal injury. Our results suggest that abdominal CT can also be used to detect early morphological changes in patients with peritoneal injury, with mural peritoneal thickening and structural changes in the omentum being the main features of imaging presentation of progressive peritoneal injury. The peritoneal mean thickness of PD patients was found to be positively correlated with dialysis age, which is consistent with the results of this study. Similar results were found for the effect of glucose exposure accumulation in the peritoneal dialysis fluid on the omental structure in relation to dialysis age. In contrast, the accumulation of sugar exposure did not significantly alter the imaging of the mural peritoneum, which may be due to the difference in sensitivity of the mural peritoneum and the omentum of high sugar stimulation. Peritonitis is a serious complication of peritoneal dialysis that results in an accelerated process of peritoneal injury due to direct damage from acute inflammation and local release of cytokines (e.g., TGF-*β*, vascular endothelial growth factor (VEGF)). The application of ultrasound to study the peritoneum revealed a positive correlation between peritoneal thickness and the development of peritonitis. The results of this study also further confirmed the effect of peritonitis on peritoneal thickening, as shown in Figure 6. Peritonitis and its severity were also noted to be independent risk factors for peritoneal thickening and omental structural abnormalities by multifactorial regression analysis.

Several studies on the application of ultrasound to the peritoneum have reported a correlation between mural peritoneal thickness and peritoneal transit function. In this study, it was found that patients with high peritoneal transit and high mean transit were more likely to have abnormal omental structure and a higher percentage of patients with wall peritoneal thickening than patients with low mean and low transit, as shown in Figure 7 but did not reach statistical significance, which may be related to the fact that the number of cases in this study is still small. This study also has some limitations, such as the small number of cases and a cross-sectional, single-center design, which may limit the generalizability of the findings, and we will next expand the study sample size and continue follow-up. Second, conducting a study on the correspondence between peritoneal CT and pathology will help to further establish the predictive value of peritoneal CT on peritoneal morphology and function. In conclusion, mural peritoneal thickening and structural changes of the omentum in patients on peritoneal dialysis are the main imaging features of progressive peritoneal injury, and peritonitis is the main risk factor for progressive peritoneal injury. CT examination of the peritoneal cavity can provide a comprehensive understanding of the characteristics and extent of peritoneal injury in peritoneal dialysis, which can help to diagnose peritoneal injury at an early stage and also provide a basis for prevention or early intervention.

This article uses single-factor and multifactor Cox regression analysis to select clinical factors related to OS. The results showed that TNM staging and CREA are independent predictors of OS, and both are risk factors for patients with OS (HR of TNM: 2.912, 95% CI, 2.188–3.875; HR of CREA: 1.020, 95% CI, 1.004–1.036). A clinical nomogram composed of TNM staging and CREA was constructed based on multivariate Cox regression analysis. The imaging omics nomogram is constructed by Rad-score and the independent clinical predictors selected above. The three predictors are all risk factors for the patient's OS (Rad-score HR: 277.920, 95%CI, 26.039–2966.297.

The calibration curve shows that there is good agreement between the clinical nomogram and radiomic nomogram to predict the survival probability of 3 and 5 years and the observation results.  Figure 8 lists the TNF-*α* and MMP-9-index values of the two nomograms. In the training set, the C-index of the clinical nomogram was 0.803 (95% CI: 0.705–0.899), and the C-index of the imaging nomogram after the Rad-score was 0.884 (95% CI: 0.808–0.940). The predictive power of the two is statistically different (*P* < 0.05). This result was verified in the validation set (imaging nomogram C-index: 0.859; clinical nomogram C-index: 0.787; *P* < 0.05). The above results show that Rad-score has gain value in predicting the OS of cc RCC. In addition, based on the imaging omics nomogram to predict the patient's 3-year and 5-year survival probability, risk grouping was used as a predictor to draw a Kaplan–Meier survival curve. There is a statistical difference between the Nomo-predicted high-risk group and the Nomo-predicted low-risk group in the training set and validation set (*P* < 0.001, log-rank test). The predicted results are consistent with the Kaplan–Meier survival analysis results of the actual survival group and the death group.

With today's artificial intelligence (AI) being paid more and more attention, the diagnostic models constructed by machine deep learning (deep learning, DL) technology represented by a convolutional neural network (CNN) have also made some progress in diagnosing renal tumors, including the differential diagnosis of the histological features of renal tumors and the research on the histological features of tumor-related genes. In the future, the Bosniak classification of renal cysts and the differential diagnosis of various rare renal subtypes by imaging histology will be our research direction, and the genomic characteristics of different metastatic cancers to predict the origin of metastasis is also a great advantage of imaging histology to predict metastasis. We believe that AI technology will be useful in image analysis in the future and will become a powerful tool for imaging physicians to diagnose diseases, which will change the future work pattern of imaging physicians. We believe that AI technology will become a powerful tool for diagnosing diseases and will change the future work pattern of imaging physicians.

## 6. Conclusion

This paper needs to show that the 10-year survival rates for grades I–IV cc RCC are 81.0%, 56.6%, 30.1%, and 18.8%, respectively. Less invasive treatments such as native nephrectomy, ablation, or even active monitoring are usually performed for low-grade cc RCC to maximize the preservation of renal units, while radical nephrectomy is required for high-grade cc RCC. Therefore, preoperative clarification of the pathologic grading of cc RCC is crucial for prognosis and selection of surgical options. Fuhrman grading obtained by puncture biopsy is the gold standard, but there are inevitable sampling errors that make an accurate preoperative assessment of the bioinvasiveness of cc RCC histopathologically challenging. Intensive CT scans are routinely performed in patients with RCC, but reliance on conventional imaging analysis does not yield information on tumor pathologic grading. The advent and rapid development of imaging histology enables automated high-throughput extraction of quantitative features of images to be informed of kidney tumors that may be overlooked or unrecognized by the naked eye. Imaging histology has made tremendous advances in technologies that meet clinical requirements and facilitate diagnosis and cancer treatment. Most of the current imaging histology studies on cc RCC are devoted to texture feature data processing and analysis at the largest tumor level, and there are limited imaging histologies for prognostic prediction analysis. Therefore, the main objective of this study is to investigate the application of 3D imaging features based on enhanced CT in the prognosis prediction of cc RCC.

## Figures and Tables

**Figure 1:** CT perfusion scan.

**Figure 2:** CT imaging features construction.

**Figure 3:** Emergency initiation of renal dialysis.

**Figure 4:** Proportion of abnormalities in retinal structure.

**Figure 5:** Independent risk factors for abnormal retinal structure.

**Figure 6:** Effect of peritonitis on peritoneal thickening.

**Figure 7:** Comparison of wall peritoneal thickening.

**Figure 8:** TNF-*α* and MMP-9-index values of the two nomograms.

## Data Availability

The data used to support the findings of this study are available from the corresponding author upon request.
